# Comparison of PLIF and TLIF in the Treatment of LDH Complicated with Spinal Stenosis

**DOI:** 10.1155/2022/9743283

**Published:** 2022-03-26

**Authors:** Xinbo Fang, Mingjie Zhang, Lili Wang, Zhengke Hao

**Affiliations:** ^1^Department of Neurosurgery, Zibo Central Hospital, Zibo 255000, China; ^2^Department of Orthopaedics and Traumatology, Qingdao Hospital of Traditional Chinese Medicine, Hiser Medical Group of Qingdao, Qingdao 266033, China; ^3^Department of Critical Care Medicine, The Affiliated Qingdao Central Hospital of Qingdao University, The Second Affiliated Hospital of Medical College of Qingdao University, Qingdao 266042, China; ^4^Department of Orthopeadic Surgery, Caoxian People's Hospital, Heze 274400, China

## Abstract

**Objective:**

The purpose was to compare the clinical effects of posterior lumbar interbody fusion (PLIF) and transforaminal lumbar interbody fusion (TLIF) in the treatment of lumbar disc herniation (LDH) complicated with spinal stenosis.

**Methods:**

96 LDH patients complicated with spinal stenosis treated in our hospital (April 2018–April 2020) were chosen as the subjects, and split into the PLIF group and the TLIF group according to different surgical approaches, with 48 cases in each group. The clinical effects of the two groups were compared.

**Results:**

There was no significant difference in hospitalization time between the two groups (*P* > 0.05). Compared with the PLIF group, the TLIF group had obviously shorter operation time and greatly lesser intraoperative blood loss (*P* < 0.05). The Numerical Rating Scale (NRS) scores of lower limb pain and low back pain in the two groups at 3 months after surgery were significantly lower than those before surgery (*P* < 0.001). The Japanese Orthopaedic Association (JOA) scores of the two groups at 3 months after surgery were significantly higher than those before surgery (*P* < 0.001). The Spitzer Quality of Life Index (SQLI) scores of the two groups at 3 months after surgery were significantly higher than those before surgery (*P* < 0.001).

**Conclusion:**

The two surgical approaches have similar efficacy in treating LDH complicated with spinal stenosis. However, PLIF is better than TLIF in terms of operation time and intraoperative blood loss, which should be adopted as the preferred surgical scheme.

## 1. Introduction

Lumbar disc herniation (LDH) is a common disease in spinal surgery that mostly occurs in the middle-aged and elderly and is predominantly in males, with main clinical manifestations such as sciatica, low back pain, and cauda equina syndrome [1, 2]. Lumbar disc is composed of annulus fibrosus, nucleus pulposus, and cartilage plate. The pathogenesis of LDH is a syndrome caused by lumbar disc degeneration, partial or total rupture of the annulus fibrosus, and stimulation or compression on the cauda equina nerve and nerve root caused by herniation of the nucleus pulposus. In addition, LDH is also related to cumulative damage, pregnancy, genetic factors, and congenital development abnormalities. Mechanical compression and inflammatory stimulation are the factors leading to lumbocrural pain in patients with LDH [3, 4]. Spinal stenosis, a common complication of LDH, refers to any form of stenosis involving the nerve root canals, spinal canals, and intervertebral foramen caused by any factors, which leads to corresponding clinical manifestations. The water content of the intervertebral disc gradually decreases with advancing age, while the cracks on its surface cause herniation of the nucleus pulposus, which compresses the nerve and spinal cord, seriously affecting the quality of life of patients. Nonoperative treatment is often adopted in LDH complicated with spinal stenosis, while operative treatment is conducted in severe cases. Most patients are relieved or cured after conservative treatment, and surgical treatment can effectively restore the nerve conduction function of patients, alleviate low back pain, promote the recovery of lumbar function, relieve lumbar spasm, restore vasoconstriction function, and improve microcirculation [5]. Recently, as the clinical spinal treatment techniques continue to improve, PLIF and TLIF have become common surgical approaches for the clinical treatment of LDH complicated with spinal stenosis, both of which have achieved significant advantages in clinical application [6]. However, there are few reports on the comparison of the therapeutic effects of the two methods. On this basis, to further investigate the clinical utility of PLIF and TLIF in the treatment of LDH patients with spinal stenosis, to provide the best treatment option for this type of patients, to reduce their clinical symptoms, and improve their life quality and prognosis.

## 2. Materials and Methods

### 2.1. General Information

96 LDH patients complicated with spinal stenosis treated in our hospital (April 2018–April 2020) were chosen as the subjects, and split into the PLIF group and the TLIF group according to different surgical approaches, with 48 cases in each group. The PLIF group had 27 males and 21 females, with an average age of 64.21 ± 3.41 years and an average disease course of 2.63 ± 0.82 years. The TLIF group had 25 males and 23 females, with an average age of 64.32 ± 3.38 years and an average disease course of 2.59 ± 0.78 years. There was no significant difference between groups in general data (*P* > 0.05).

### 2.2. Inclusion Criteria

The inclusion criteria were as follows: (1) the patients met the diagnostic criteria of LDH complicated with spinal stenosis in the 12th edition of *Campbell's Operative Orthopaedics* [7] and confirmed by imaging examination [2]; the efficacy was poor after 6 months of conservative treatment [3]; and this study as approved by the hospital ethics committee, and all patients signed the informed consent.

### 2.3. Exclusion Criteria

The exclusion criteria were as follows: (1) the patients were complicated with immune system diseases [2]; the patients had spinal instability and intervertebral disc inflammatory lesions [3]; and the patients had confusion and mental and other cognitive disorders.

### 2.4. Methods

Patients in the PLIF group were treated with PLIF. The supine position was taken, and the specific lesions were examined with the assistance of the C-arm machine. Then, a median longitudinal incision was made, and the incised tissue was separated to both sides. After positioning, the pedicle screw was placed. Then, the ligaments in the interspace related to the lesions were cut off and some ligaments were removed. The nerve root decompression was adopted, the contralateral traction was carried out, and the diseased intervertebral disc tissue was removed. After the abovementioned operations, the intervertebral space was rinsed, bone fragments were placed under longitudinal pressure, the screw cap was tightened, and the fixed position and effect were determined. The negative pressure drainage tube was placed after the wound was rinsed, and then the wound was sutured.

Patients in the TLIF group received TLIF. The supine position was taken, and the body surface projections of the L3, L4, and L5 pedicles were located under fluoroscopy. The skin was cut and a guiding needle was inserted into the middle part of the L3 and L4 right facet joints. After further expansion, a working tube was placed. The bone knife was used to remove part of the L3 inferior joint protrusion and L4 superior joint protrusion to expose the L4 nerve root and the L3/4 intervertebral disc. The intervertebral disc tissue was removed, and the upper and lower cartilage endplate tissues were scraped. The cage was implanted through the intervertebral foramen. The same method was used for L4/5. Under fluoroscopy, the pedicle guide wires were tapped along the right the L3, L4, and L5, and 3 Voyager screws were inserted. The left side was cut 1–2 cm on the body surface according to the body surface projections of the L3, L4, and L5 pedicles. The guide wires were inserted under fluoroscopy, the casing was inserted step by step, and three Voyager screws were inserted, respectively. The position of the cage and screw was confirmed by X-ray after surgery.

Antibiotics, dehydrating agents, and neurotrophic drugs were used in both groups after surgery, and the drainage tube was removed according to the clinical conditions of the patients 48 hours after surgery. Support was worn to assist activities 3 days after operation, and the cycle was 3 months. Heavy physical labor was avoided during the period [8].

### 2.5. Evaluation Indexes

Patients' clinical indicators of the two groups were recorded and counted, including operation time, intraoperative blood loss, and hospitalization time.

The Numerical Rating Scale (NRS) [9] was used to evaluate the degree of lower limb pain and low back pain of patients in the two groups before surgery and 3 months after surgery. A higher score indicated more serious pain of patients.

The Japanese Orthopaedic Association Scores (JOA) [10] was used to evaluate the improvement of lumbar function in the two groups before surgery and 3 months after surgery. A higher score indicated better improvement of lumbar function.

Spitzer Quality of Life Index (SQLI) [11] was used to evaluate the life quality of patients in the two groups before surgery and 3 months after surgery. Higher score indicated better life quality.

### 2.6. Statistical Methods

All the experimental data were collected by SPSS 21.0 software for statistical analysis and processing, and the data are plotted by GraphPad prism 7 (GraphPad software, San Diego, USA). The count data were tested by *χ*^2^, expressed by (*n* (%)), and the measurement data were measured by the *t*' test, expressed by ($\bar{x}\pm s$). The difference was statistically significant when *P* < 0.05.

## 3. Results

### 3.1. Between-Group Comparison of Clinical Indicators

There was no significant difference in the length of hospital stay between groups (*P* > 0.05). Compared with the PLIF group, the TLIF group had obviously shorter operation time and greatly less intraoperative blood loss (*P* < 0.05; Table 1).

### 3.2. Between-Group Comparison of Perioperative Scores

The NRS scores of lower limb pain and low back pain 3 months after the operation were significantly lower than those before the operation (*P* < 0.05). The JOA scores of the two groups at 3 months after surgery were significantly higher than those before surgery (*P* < 0.001; Figure 1).

### 3.3. Comparison of SQLI Scores before Surgery and 3 months after Surgery between the Two Groups

The SQLI scores of the two groups at 3 months after surgery were significantly higher than those before surgery (*P* < 0.05; Figure 2).

## 4. Discussions

Lumbar vertebrae are the key positions of torso activity, and any activity will increase the burden of lumbar vertebrae. Therefore, LDH will become more obvious and serious in the case of long-term heavy physical labor, with early manifestations such as recurrent lumbocrural pain, lower limb radioactive pain, numbness, and weakness. LDH is an important factor in inducing spinal stenosis. In recent years, since the understanding of the spinal structure and the in-depth exploration of biomechanics have greatly promoted the progress of spinal surgery technology, PLIF and TLIF have attracted much attention in the treatment of LDH complicated with spinal stenosis [12]. PLIF can well expose the nerve root without affecting the blood supply of the graft, promote the recovery of intervertebral space height, and maintain the integrity of the posterior joints. Posterior intervertebral bone grafting is performed while directly observing the nerve root and the dural sac with high safety [13]. TLIF can achieve intervertebral decompression and fusion under direct vision, so that the spine is stable, with less damage to the lumbar structure and less amount of intraoperative blood loss [14]. However, it is worth noting that the correct placement of the expansion channel is the key to the success of the surgery. Therefore, the center of the pedicle should be correctly located before surgery. When stripping the soft tissue of the upper and lower facet joints, it should be close to the bone and not exceed the lateral edge of the facet joints so as not to damage the outlet branches of nerve roots and vascular bundles. For limited visual field of operation under the channel, fluoroscopy should be performed several times in percutaneous screw placement so that the direction of the screws is not deviated [15].

This study showed that the NRS scores of lower limb pain and low back pain in the two groups after surgery were significantly lower than those before surgery (*P* < 0.001), suggesting that the two surgical approaches can greatly ease the limb pain of LDH patients complicated with spinal stenosis, which is conducive to disease treatment. In addition, the SQLI scores of the two groups after surgical treatment were significantly higher than those before treatment. Ilyas et al. [16] pointed out in their study that after PLIF and TLIF were performed for patients with lumbar degenerative diseases, the SQLI scores of the PLIF group (7.23 ± 0.64) and the TLIF group (7.31 ± 0.58) at 6 months after surgery were significantly higher than (4.95 ± 0.82) and (4.86 ± 0.76) before surgery, indicating that both surgical approaches can improve the life quality of patients and the prognosis.

In conclusion, the efficacy of the two surgical approaches in the treatment of lumbar disc herniation complicated with spinal canal stenosis is similar. However, TLIF is superior to TLIF in terms of operation time and intraoperative blood loss and should be the first choice.

## Figures and Tables

**Figure 1:** Comparison of perioperative scores between the two groups ($\bar{x}\pm s$). Note: (a) Comparison of lower limb pain NRS scores before surgery and 3 months after surgery between the two groups. The abscissa represents before surgery and 3 months after surgery, and the ordinate represents NRS score of lower limb pain (points). The lower limb pain NRS scores in PLIF group were (6.73 ± 0.81) and (1.64 ± 0.32) before surgery and 3 months after surgery, respectively. The lower limb pain NRS scores in TLIF group were (6.69 ± 0.79) and (1.68 ± 0.28) before surgery and 3 months after surgery, respectively. ^*∗*^indicated a significant difference in the lower limb pain NRS scores of the PLIF group before surgery and 3 months after surgery (*t* = 40.491, *P* ≤ 0.001); ^*∗∗*^indicated a significant difference in the lower limb pain NRS scores of the TLIF group before surgery and 3 months after surgery (*t* = 41.413, *P* ≤ 0.001). (b) Comparison of low back pain NRS scores before surgery and 3 months after surgery between the two groups. The abscissa represents before surgery and 3 months after surgery, and the ordinate represents NRS score of low back pain (points); The low back pain NRS scores in PLIF group were (5.46 ± 1.53) and (1.52 ± 0.46) before surgery and 3 months after surgery, respectively. The low back pain NRS scores in TLIF group were (5.48 ± 1.49) and (1.56 ± 0.4) before surgery and 3 months after surgery, respectively. ^*∗*^indicated a significant difference in the low back pain NRS scores of the PLIF group before surgery and 3 months after surgery (*t* = 17.086, *P* ≤ 0.001); ^*∗∗*^indicated a significant difference in the low back pain NRS scores of the TLIF group before surgery and 3 months after surgery (*t* = 17.513, *P* ≤ 0.001). (c) Comparison of JOA scores before surgery and 3 months after surgery between the two groups. The abscissa represents before surgery and 3 months after surgery, and the ordinate represents JOA scores (points); The JOA scores in PLIF group were (15.23 ± 4.31) and (22.15 ± 1.45) before surgery and 3 months after surgery, respectively. The JOA scores in TLIF group were (15.26 ± 4.36) and (22.43 ± 1.54) before surgery and 3 months after surgery, respectively. ^*∗*^indicated a significant difference in the JOA scores of the PLIF group before surgery and 3 months after surgery (*t* = 10.543, *P* ≤ 0.001); ^*∗∗*^indicated a significant difference in JOA scores of the TLIF group before surgery and 3 months after surgery (*t* = 10.743, *P* ≤ 0.001).

**Figure 2:** Comparison of SQLI scores before surgery and 3 months after surgery between the two groups ($\bar{x}\pm s$). The abscissa represents before surgery and 3 months after surgery, and the ordinate represents SQLI scores (points); The SQLI scores in PLIF group were (5.03 ± 0.82) and (7.34 ± 0.65) before surgery and 3 months after surgery, respectively. The SQLI scores in TLIF group were (5.06 ± 0.74) and (7.41 ± 0.58) before surgery and 3 months after surgery, respectively. ^*∗*^indicated ta significant difference in the SQLI scores of the PLIF group before surgery and 3 months after surgery (*t* = 15.295, *P* ≤ 0.001); ^*∗∗*^indicated a significant difference in SQLI scores of the TLIF group before surgery and 3 months after surgery (*t* = 17.317, *P* ≤ 0.001).

**Table 1:** Comparison of clinical indicators between the two groups ($\bar{x}\pm s$).

Group	*n*	Operation time (min)	Intraoperative blood loss (mL)	Hospitalization time (d)
PLIF group	48	138.73 ± 12.34	608.28 ± 36.72	17.82 ± 4.27
TLIF group	48	106.24 ± 13.42	375.24 ± 31.52	17.86 ± 4.31
*T*		12.347	33.363	0.047
*P*		≤0.001	≤0.001	0.964

## Data Availability

The datasets used and/or analyzed during the present study are available from the corresponding author on reasonable request.
